This article has been retracted.

# Inhibitory potentials of *Streptomyces exfoliatus* strain ‘MUJA10’ against bacterial pathogens isolated from rural areas in Riyadh, Saudi Arabia

**DOI:** 10.1371/journal.pone.0266297

**Published:** 2022-04-14

**Authors:** Jawaher Ibrahim Alahadeb

**Affiliations:** Department of Biology, College of Education (Majmaah), Majmaah University, ALmajmaah, Saudi Arabia; Mendel University of Agriculture and Forestry: Mendelova univerzita v Brne, CZECH REPUBLIC

## Abstract

Healthcare-associated infections are resulting in human morbidity and mortality worldwide. These infections are directly proportional to increased multidrug resistance (MDR), which limits antibiotic treatment and make the treatment of infections challenging. *Streptomyces* spp. are well known to produce various biologically active compounds. Therefore, these are considered as promising biological control agents against wide range of bacterial pathogens. This study was conducted to isolate and identify the most efficient antibiotic-producing *Streptomyces* St 45 isolate against *Staphylococcus aureus* ATCC29737, *Salmonella typhimurium* ATCC25566, *E*. *coli* 0157h7 ATCC25922 and *Bacillus subtilis*. A total 40 soil and 10 water (from wells) samples were processed using standard microbiological techniques at King Faisal Research Centre, Riyadh, Saudi Arabia. The selected *Streptomyces* St 45 isolate was grown to produce biologically active metabolites, and the minimum concentration (MIC) was determined. Sixty isolates with antibacterial properties were selected. The 16s rRNA gene analysis was used to identify the strongest *Streptomyces* St 45 strain. The highest zone of inhibition (ZOI) was provided by ‘MUJA10’ strain of *S*. *exfoliatus* against *Staphylococcus aureus* ATCC29737 (51.33 ± 2.15 mm). The MIC value of ‘MUJA10’ metabolite of *S*. *exfoliatus* strain against *Salmonella typhimurium* ATCC25566 and *E*. *coli* 0157h7 ATCC25922 was 0.125 mg/ml. However, *Bacillus subtilis* had a MIC of 0.625 mg/ml and *Staphylococcus aureus* ATCC29737 had a MIC of 2.5 mg/ml. In conclusion, *Streptomyces exfoliatus* strain ‘MUJA10’ obtained from soil exhibited high inhibitory potential against human pathogens. The 16s rRNA gene analysis revealed that *Streptomyces* St 45 isolate was similar to *Streptomyces exfoliatus* A156.7 with 98% similarity and confirmed as *Streptomyces exfoliates* ‘MUJA10’ at gene bank with gene accession number OL720257.

## Introduction

Multidrug resistance (MDR) in bacterial pathogens is regarded as a global health challenge and represents a serious problem for public health leading to high mortality in human [1–4]. Globalization, overuse of antibiotics, and self-medication are the most responsible factors spreading antibiotic resistance [5, 6]. Several studies have predicted that no effective antibiotic will be available to treat infectious diseases till 2050 because of increasing pathogenic antibiotic resistance [7–10]. Many bacterial species have become multi-drug resistant, and Colistin-resistant *Enterobacter*, and *Klebsiella pneumoniae*, Fluoroquinolone-resistant *Escherichia coli*, third generation cephalosporin-resistant *Neisseria gonorrhoeae*, and Methicillin-resistant *Staphylococcus aureus* (MRSA) are being focused in recent research [11–14]. Human pathogens such as carbapenem-resistant *Acinetobacter baumannii*, *Pseudomonas aeruginosa*, and *Enterobacteriaceae* are listed as the highest priority species [15,16]. Similarly, Vancomycin-resistant Enterococci, MRSA, Fluoroquinolone-resistant Salmonella, Campylobacter, and Shigella are considered as multidrug resistant pathogens [13]. Therefore, discovery and development of new antibiotics are urgently needed to solve drug resistance problem [6]. *Streptomyces* belongs to Streptomycetaceae family in the order Actinomycetales and class Schizomycetes [17]. These are found in soils, manure, and other sources [18,19]. These are eubacteria and grow by forming filaments or mycelium and do not form the usual bacterial assembly as bacillary or coccoid forms [20]. They produce chained conidiospores from spore-bearing aerial hyphae. All *Streptomyces* spp. are Gram-positive, their colony structure is complex according to the presence of multinucleate, shape of branching mycelia and the formation of vegetative and reproductive colony structures [21].

Soil is one of the richest sources of bacteria and actinomycetes. *Streptomyces* is one of the most important genera because of their major diversity and proven ability to produce novel bioactive compounds. The produced compounds serve as antifungal, antiviral, antitumor, and antihypertensive agents, immunosuppressant, and particularly antibiotics [22,23]. Baltz [24] reported that out of 1025 *Actinomycetes* isolates in 1 gm of soil, 105 have been isolated and screened for antibiotics production in the last 50 years. Nevertheless, *Streptomyces* produce about 70% of the world’s naturally occurring antibiotics [25,26]. *Streptomyces*’s biodiversity is considered as one of the most important parameters for screening of new antibiotics. *Streptomyces* are known to produce different types of antibiotics namely peptide/glycopeptides, angucyclinone, tetracyclines, phenazine, macrolide, anthraquinone, polyene, nonpolyene, benzoxazolophenanthridine, heptadecaglycoside, lactones and others.

Amid successful trials for discovering new sources and alternatives for antibiotics, infectious diseases remained the second leading cause of death worldwide. Bacterial infections cause about 17 million deaths annually, mainly in children and elder persons. Therefore, this study was aimed at isolating new strains of antibiotic producing *Streptomyces* sp. and to test their inhibitory activities against some bacterial pathogens.

## Materials and methods

### Ethics statement

The written consent was taken from the participants and the institutional ethics committee of Majmaah University approved this study.

### Microorganisms and media

All human bacterial pathogens were obtained from King Faisal Research Centre, Riyadh, Saudi Arabia. All media were prepared as described by APHA [27]. Starch and casein agar was used for isolation and maintenance of *Streptomyces* sp. isolates. It consisted of (g/l): casein 1, starch 10 and agar 15. Muller Hinton agar was used for determining the inhibitory activity of *Streptomyces* sp. isolates against bacterial strains. It contained beef, dehydrated infusion 30.0, casein hydrolysate 17, Starch 1.5, agar 15.0 with pH adjusted to 7.2 ± 0.1 at 25 °C.

### Soil and water sampling for *Streptomyces* sp. isolates

A total 40 soil samples and 10 water samples (wells’ water) were collected from rural areas at different geographical locations in Riyadh, Saudi Arabia. Soil samples were collected at depth of 10 cm and packed in sterilized glass jars, transported to the lab, and stored at 4°C for further use [28]. Water samples were collected from wells in different locations in Riyadh. Before obtaining water samples, water was left to run for 10 minutes, then 100 ml sample was collected in sterilized glass jars, transported to the lab, and stored at 4°C for more further studies. Isolation was done by inoculating starch and casein agar plates with soil and water samples individually and the plates were incubated at 30°C for 3–5 days. Rough colonies were picked up and streaked on starch and casein agar. The colonies were stored at 4°C and sub-cultured at monthly intervals.

### Standard inoculum

Five ml of peptone water were inoculated by 3–5 single colonies of the selected isolate and incubated at 37 °C for 24 h. Thereafter, optical density (OD) of the culture was adjusted to 0.06–0.8 using the spectrophotometer at 625 nm which is equivalent to (14×10^6^ CFU/ml) to prepare the standard inoculum [29].

### Morphological characteristics of the selected isolates

Colony color and gram staining were examined microscopically for studying the morphological features. All morphological characters were carried out in triplicates.

### Inhibitory potential of *Streptomyces* isolates against the growth of pathogenic bacteria

Disc diffusion method was done to test the inhibitory potentials of *Streptomyces* isolates against *Staphylococcus aureus* ATCC29737, *Bacillus subtilis*, *Salmonella typhimurium* ATCC25566 and *E*. *coli* 0157h7 ATCC25922 according to the Kirby-Bauer agar disc diffusion method [25]. The plates were incubated at 30 ºC for 3–5 days and clear zones around the discs were measured in mm. The most significant strain showing the antibacterial properties was grown in starch and casein broth under the optimal conditions of 30°C and 150 rpm for 5 days. The biologically active metabolites were extracted by centrifugation at 10000 rpm for 15 minutes. The pellets were discarded, and the supernatant was collected for further studies. The extract was subjected to secondary screening against *Staphylococcus aureus* ATCC29737, *Bacilllus subtilis*, *Salmonella typhimurium* ATCC25566 and *Escherichia coli* 0157h7 ATCC25922 by agar well diffusion method. Muller Hinton agar medium was poured into Petri dishes and inoculated with 1 ml of *E*. *coli*, *S*. *aureus* and *S*. *typhimurium* (14×10^6^ CFU/ml) using spreading technique. Agar wells were made using a sterilized 7 mm corkborer and filled by 100 μl of the tested supernatant. Petri dishes were incubated at 30 °C for 5 days. All experiments were carried out in triplicates. The supernatant inhibitory activity was expressed as the inhibition zone diameter’s mean [30].

### Minimum inhibitory concentration (MIC) of *Streptomyces* culture supernatant

The MIC was determined by the tube dilution method. Different concentrations of supernatant were prepared. Starch and casein broth was prepared and inoculated with 1 ml of the different supernatant concentration and incubated at 30 ºC for 5 days. The OD was measured at 625 nm. The MIC was calculated according to Tian et al. [23].

### Identification of the selected isolate using 16s rRNA

The selected isolate was further identified using phylogenetic analysis of 16SrRNA gene sequences. Isolation of cellular DNA was completed as described by Fredrick [31] and amplification of 16SrRNA was done according to Lane [32] using the two universal primers (F1: 5, AGAGTTT (G/C) ATCCTGGCTCAG 3, and R1 5, ACGG (A/C) TACCTTGTTACGACTT 3). The sequence reads were edited and assembled using Bio Edit version 7.0.4 and cluster W version 4.5.1. BLAST searches were done using the NCBI server According to Al-Dhabi et al. [33].

### Statistical analysis

The collected data were statistically analyzed on SPSS 26.0 for windows. One-way analysis of variance (ANOVA) was used to infer the significance in the dataset. The data were normally distributed; therefore, analysis was done on original data. Tukey’s HSD post-hoc test at 95% probability was used for multiple comparisons where ANOVA denoted significant differences.

## Results

### Isolation of Streptomyces isolates from soil and water samples

A total 40 soil and 10 water samples from different geographical locations of some rural areas in Riyadh, Saudi Arabia were subjected to isolation of actinomycetes. Sixty (60) different actinomycetes exhibiting antimicrobial properties were separated based on pigmentation (Fig 1). All obtained isolates were filamentous and positive for gram staining (Fig 2). Actinomycetes strains producing dark beige pigments were the most predominant.

**Fig 1:** Morphological characters of *Streptomyces* sp. isolates according to their pigment production.

**Fig 2:** Morphological characters of *Streptomyces* sp. isolates according to Gram staining.

### Inhibitory activity of Streptomyces isolates against Gram-positive and Gram-negative bacterial pathogens

All isolates were tested for the inhibitory activities against four pathogenic bacteria *E*. *coli* and *Salmonella typhymurium* (as Gram negative bacteria) and *Bacillus subtilis*, *Staphylococcus aureus* as (Gram positive bacteria) using disc diffusion test. Ten of these isolates exhibited inhibitory activity against only Gram positive bacteria, 42 isolates inhibited only Gram negative bacteria and 8 isolates inhibited both Gram positive and Gram negative bacteria. The most potent isolate was selected as shown in Table 1.

**Table 1:** Number of bioactive actinomycetes isolates with inhibitory activity against pathogenic bacteria.

Colony color	G +ve only	G -ve only	Both G +ve and G -ve
Dark beige	0	2	0
Light beige	1	2	0
Dirty white	1	10	2
white	1	10	4
Grey	3	13	2
Dark green	0	4	0
Green	4	1	0
Red	0	1	0
Pink	0	1	0

### Antimicrobial activity of bioactive compounds using disc diffusion test

Antimicrobial activity of bioactive compounds in culture supernatant is shown in Fig 3. *Streptomyces exfoliatus* strain ‘MUJA10’ showed the highest antimicrobial activity against *Staphylococcus aureus* (51.33±3.02 mm), followed by *E*. *coli* (33.55±2.08 mm). The lowest inhibitory activity was recorded for *Salmonella typhumurium* (28.60±3.06 mm) and *Bacillus subtilis* (25.55±3.08 mm).

**Fig 3:** Antimicrobial activity of bioactive compounds of *Streptomyces exfoliatus* strain ‘MUJA10’ against *Staphylococcus aureus*, *E*. *coli*, *Salmonella typhumurium* and *Bacillus subtilis*.

### Minimal inhibitory concentration of *Streptomyces exfoliatus* MUJA10 strain against bacterial pathogens

In MIC evaluation of bioactive compound, *Streptomyces exfoliatus* strain ‘MUJA10’ exhibited the lowest values against all test organisms 0.125mg/ml for *E*. *coli* and *Salmonella typhimurium*, 0.625 mg/ml for *Bacillus subtilis*, 2.5 mg/ml for *Staphylococcus aureus* (Fig 4).

**Fig 4:** Minimal inhibitory concentration of *Streptomyces exfoliatus* strain ‘MUJA10’ against *Staphylococcus aureus*, *E*. *coli*, *Salmonella typhumurium* and *Bacillus subtilis*.

### Molecular identification of Streptomyces St45 isolate using 16S rRNA genetic sequencing

The 16S r RNA was sequenced with using universal primer with an amplified product of 1500bp and obtained sequence was compared with Gen Bank databases using BLASTN software by NCBI (https://www.ncbi.nlm.nih.gov/). Similarity percentage is shown in Fig 5, where 16S rRNA sequence of the isolate *Streptomyces* St 45 revealed a close relatedness with 98% similarity. As shown in Fig 5, the phylogenetic analysis of nucleotide sequences based on 16S rRNA revealed closely to *Streptomyces exfoliates* A156.7. Hence, the strain was confirmed as *Streptomyces exfoliatus* strain ‘MUJA10’.

**Fig 5:** Phylogenetic analysis of *Streptomyces exofoliatus* MUJA10 strain isolate using 16S rRNA genetic sequencing.

## Discussion

Non-judicious use of antibiotics is the main reason for increased number of multidrug-resistant pathogens around the world [34]. Multidrug-resistant nosocomial pathogens are responsible for life-threating infections and diseases [35]. Nowadays, there is a big challenge for discovering new alternative antibiotics combating the multidrug-resistant pathogenic strains [6]. *Streptomyces* species are one of the most efficient microorganisms producing biologically active compounds [22,23]. It has been found that *Streptomyces* sp. is highly effective against many multidrug-resistant deadly pathogens [24]. Among these pathogens, *Staphylococci* and *Enterobacter* are considered the second cause for nosocomial infections after *Staphylococci*. Thereafter, Streptomyces remain remarkably effective against most ESKAPE pathogenic strains (*Enterococcu*s *faecium*, *Staphylococcus aureus*, *Klebsiella pneumoniae*, *Acinetobacter baumanni*, *Pseudomonas aeruginosa*, and *Enterobacter* sp.) [25,26]).

In this study, 60 different isolates of antibiotic producing *Streptomyces* against different Gram positive and negative bacterial pathogens were isolated from different water and soil sources. It was found that the white and grey colored *Streptomyces* isolates were the main dominant pigmented isolates. In addition, most of them are active against pathogenic gram-positive bacteria. These results are in consistent with Gautham et al. [36], who reported the advantages of white and gray *actinomycetes* with an inhibitory potential of 5% against Gram positive pathogens and 36% against Gram negative pathogens. As discovered by Fenical et al. [37], the higher susceptibility of Gram positive bacteria was due to the lack of lipopolysaccharide outer membrane. Results of the current study are similar to Singhania et al. [38], who found that *Streptomyces laurentii* VITMPS isolated from marine soil had the ability inhibit the growth of *Bacillus cereus* with inhibition zone of 35 mm and *Escherichia coli* with inhibition zone 35 mm. Singhania et al. [38] also reported that MIC of the crude extract against *Bacillus cereus* (MTCC No: 6840) and *Escherichia coli* (MTCC No: 1588) was 100 μg mL-1. The results of the current study illustrated that *Streptomyces* St 45 isolate exhibited inhibitory activity against *Staphylococcus aureus* ATCC29737 with a MIC of 2.5 mg/ml.

The results of the current study are in agreement with Junaidah et al. [39], who tested the inhibitory activity of *Streptomyces* sp. SUK 25 against methicillin-resistant *Staphylococcus aureus* and reported MIC of 2.44 ± 0.01 μg/mL, whereas the lowest reported MIC was 1.95 μg/mL based on a seven-day culture. Results of the current study showed that *Streptomyces* St 45 isolate was active against pathogenic bacteria. In contrast, Rai et al. [40] reported a low MIC value of 1 mg/ml for MRSA. Enright [41], reported that MIC value is affected by several parameters, including susceptibility of the organism, type of microorganisms, concentration and type of biologically active metabolites, composition of the medium, incubation temperature and time. *Streptomyces* St 45 isolate was identified DNA analysis and was confirmed with Gene bank records as *Streptomyces exofoliatus* MUJA 2010 with gene accession number of OL720257.

## Conclusion

In conclusion, current study showed that soil and water of some rural areas in Riyadh, Saudi Arabia contained diverse *Streptomyces* strain that can inhibit the growth of some pathogenic bacteria. Among screened isolates, *Streptomyces exfoliatus* strain ‘MUJA10’ was the most effective against tested bacterial pathogens. Further studies regarding characterization of bioactive compounds are essential.
